The article "Comparison of confirmed and probable COVID-19 patients in the intensive care unit during the normalization period" was published in 2021. Journal: Bosn J Basic Med Sci.

# Comparison of confirmed and probable COVID-19 patients in the intensive care unit during the normalization period

**DOI:** 10.17305/bjbms.2021.6657

**Published:** 2021-11-22

**Authors:** Fatma İrem Yeşiler, Mesher Çapras, Emre Kandemir, Helin Şahintürk, Ender Gedik, Pınar Zeyneloğlu

**Affiliations:** Department of Anesthesiology and Critical Care Unit, Baskent University Faculty of Medicine, Ankara, Turkey

**Keywords:** Confirmed, COVID-19, intensive care unit, normalization period, probable, SARS-CoV-2

## Abstract

The decrease in social distance together with the normalization period as of June 1, 2020, in our country caused an increase in the number of coronavirus disease 2019 (COVID-19) patients. Our aim was to compare the demographic features, clinical courses, and outcomes of confirmed and probable COVID-19 patients admitted to our intensive care unit (ICU) during the normalization period. Critically ill 128 COVID-19 patients between June 1, 2020, and December 2, 2020, were analyzed retrospectively. The mean age was 69.7 ± 15.5 y (61.7% male). Sixty-one patients (47.7%) were confirmed. Dyspnea (75.0%) was the most common symptom and hypertension (71.1%) was the most common comorbidity. The mean Acute Physiology and Chronic Health Evaluation System (APACHE II) score; Glasgow Coma Score; Sequential Organ Failure Assessment scores on ICU admission were 17.4 ± 8.2, 12.3 ± 3.9, and 5.9 ± 3.4, respectively. One hundred and one patients (78.1%) received low-flow oxygen, 48 had high-flow oxygen therapy (37.5%), and 59 (46.1%) had invasive mechanical ventilation. Fifty-three patients (41.4%) had vasopressor therapy and 30 (23.4%) patients had renal replacement therapy due to acute kidney injury (AKI). Confirmed patients were more tachypneic (*p* = 0.005) and more hypoxemic than probable patients (*p* < 0.001). Acute respiratory distress syndrome and AKI were more common in confirmed patients than probable (both *p* < 0.001). Confirmed patients had higher values of hemoglobin, C- reactive protein, fibrinogen, and D-dimer than probables (respectively, *p* = 0.028, 0.006, 0.000, and 0.019). The overall mortality was higher in confirmed patients (*p* = 0.209, 52.6% vs. 47.4%). Complications are more common among confirmed COVID-19 patients admitted to ICU. The mortality rate of confirmed COVID-19 patients admitted to the ICU was found to be higher than probable patients. Mortality of confirmed cases was higher than prediction of APACHE-II scoring system.

## INTRODUCTION

Coronavirus disease 2019 (COVID-19) is defined as a contagious disease caused by severe acute respiratory syndrome (SARS). On December 31, 2019, the first case of pneumonia was reported in Wuhan, China’s Hubei province, and on January 31, 2020, the World Health Organization declared the new coronavirus infection, called COVID-19, as a global pandemic [1,2].

This virus has the characteristics of the beta-coronavirus subgroup from the Coronavirus family. It is transmitted by droplet and contact. It is noticed that the contamination can start 1-2 days before the symptoms and continue until the 14^th^ day after the symptoms. Symptomatic patients with COVID-19 may experience severe pneumonia, respiratory failure (acute respiratory distress syndrome [ARDS]), and/or organ dysfunctions (etc., sepsis, septic shock, acute cardiac injury, acute renal injury) [3,4]. Intubation, mechanical ventilation (MV), and intensive care unit (ICU) follow-up may be required [3-5]. About 14% of COVID-19 cases are severe and 5% are critical [6].

Real-time polymerase chain reaction (RT-PCR) is the gold standard method for the diagnosis of COVID-19. Infected or symptomatic patients may have negative results due to technical reasons such as poor quality sample with little material, testing at early or late stage of infection, proper sample handling, PCR inhibition or virus mutation, and fluctuating distribution of the virus in symptomatic and asymptomatic cases [7,8]. Therefore, probable cases are considered to be patients with a low viral load or where the range of viral transmission is difficult to detect.

On March 11, 2020, the first confirmed COVID-19 patient was declared in Turkey [5]. During the COVID-19 pandemic, the Ministry of Health dedicated it as a normalization period as of June 1, 2020 [8]. The decrease in social distance together with the normalization period in our country caused an increase in the number of daily tests and overall confirmed cases.

We planned this study due to the lack of data on the comparison of confirmed and probable COVID-19 patients admitted to the ICU. Our aim was to compare the demographic and clinical features, complaints, comorbidities, intubation-MV requirement, treatments, complications, clinical courses, and outcomes of confirmed and probable COVID-19 patients admitted to our ICU during the normalization period.

## MATERIALS AND METHODS

### Study design and participants

The medical records of patients aged 18 years or more with confirmed and probable COVID-19 from June 1, 2020, to December 2, 2020, were retrospectively analyzed at our center. Patients younger than 18 years, whose data were not available and who were not admitted with confirmed or probable diagnosis of COVID-19 were excluded from the study.

Probable case was defined as a patient with a negative COVID-19 RT-PCR who had symptoms, risk factors, and/or radiological findings. Confirmed case was identified as a patient with a positive COVID-19 PCR [8,9].

The primary outcome of the study is to determine and compare the incidence of confirmed and probable critically ill COVID-19 patients, the need for intubation-MV, and ICU-hospital mortality. The secondary outcome is to compare the complications, laboratory results, length of ICU, and hospital stay between confirmed and probable critically ill COVID-19 patients.

### Data collection

The following data were obtained from electronic medical and nursing records: Patient age; sex; complaints; exposure and travel history; comorbidities; Acute Physiology and Chronic Health Evaluation System (APACHE II) score; Sequential Organ Failure Assessment (SOFA) score; Glasgow Coma Score (GCS); vital signs at ICU admission; microbiological sample type; PCR results; arterial blood gas analysis; need for intubation and mechanical ventilation (MV) (non-invasive or invasive); ventilation parameters (tidal volume, positive end-expiratory pressure [PEEP], and fraction of inspired oxygen [FIO_2_]), arterial partial pressure of oxygen (PaO_2_), PaO_2_/FIO_2_ ratio; prone position; renal replacement therapy (RRT); laboratory values; treatment (vasopressor agents, antiviral drugs, and corticosteroids); length of ICU-hospital stay; and ICU-hospital mortality.

### Laboratory procedures

Nasal and/or oropharyngeal swab or tracheal aspirate samples of COVID-19 patients were performed by RT-PCR assay. Laboratory examinations were complete blood count, D-dimer, coagulation profile, serum biochemical tests (renal and liver function tests, creatinine kinase, lactate dehydrogenase [LDH], and electrolytes), myocardial enzymes, ferritin, C-reactive protein (CRP), and procalcitonin (PCT). All patients underwent posterior anterior chest radiography and chest computed tomography (CT). The intensivist decided on the frequency of the examinations.

### Definitions

Probable and confirmed cases were defined according to the COVID-19 guideline of the Turkish Republic Ministry of Health. The criterion for admission to the ICU was evaluated according to the guide of the Ministry of Health [8,9]. These criteria were as follows: Patient who has dyspnea and respiratory distress; respiration rate ≥30/min, PaO_2_/FiO_2_ <300; oxygen requirement increasing in follow-up; SpO_2_ <90% or PaO_2_ <70 mmHg despite 5 L/min oxygen therapy; hypotension (systolic blood pressure <90 mmHg and 40 mmHg than usual SBP more than decrease and mean arterial pressure <65 mmHg, tachycardia >100/minute; patients with acute organ dysfunction such as acute kidney injury (AKI), acute liver failure, confusion, acute coagulopathy and immunosuppression; elevated troponin level and arrhythmia; lactate >2 mmol; and presence of skin disorders such as capillary return disorder and cutis marmaratus. All confirmed and probable critically ill COVID-19 patients were isolated on a ward of the ICU.

Fever was defined as a tympanic measurement of 37.8°C and higher. Sepsis and septic shock were defined according to the 2020 Surviving Sepsis Campaign: Guidelines on the Management of Critically Ill Adults with COVID-19 [10]. Pneumonia was diagnosed on the basis of the American Thoracic Society and Infectious Diseases Society of America criteria [11]. AKI was identified on the basis of the Kidney Disease Improving Global Outcomes (KDIGO) clinical practice guidelines [12] and ARDS was diagnosed according to the Berlin Definition [10,13]. Disseminated Intravascular Coagulation (DIC) was defined as a cumulative score of five or more from prolonged prothrombin time (PT), reduced platelets and fibrinogen, and elevated fibrin-related markers [8,14,15]. The overall mortality rate includes deaths from all causes and deaths after transfer to another hospital.

### Ethical statement

This study was approved by the Başkent University Institutional Review Board (project no: KA20/383).

### Statistical analysis

The statistical analysis was performed using the Statistical Package for the Social Sciences 25.0 (version 25.0; SPSS Inc., Chicago, IL, USA). Frequencies were expressed as numbers (n) and percentages (%). Variables are expressed as mean values ± standard deviation. Categorical variables between the two groups were analyzed with the Chi-square test. The non-parametric continuous variables between confirmed and probable groups were compared by Mann–Whitney test. *p* < 0.05 was considered statistically significant.

## RESULTS

During the period, 342 patients were admitted to ICU and 128 of them were diagnosed with COVID-19. Sixty-one patients of 128 patients (47.7%) were confirmed and 67 patients (52.3%) were probable (Figure 1). Out of 128 COVID-19 patients, 79 (61.7%) were male. The mean age of all patients was 69.7 ± 15.5 years (between 23 and 95 years). Most of the patients (96.1%, n: 123) were admitted from the emergency and other wards within our hospital. Sixty-two patients (48.4%) had medical etiologies and 66 patients (51.6 %) had surgical causes. There were 7 renal (5.5%) and 3 liver (2.3%) transplant recipients. Dyspnea (75.0%) was the most common symptom and hypertension (71.1 %) was the most common comorbidity. Confirmed patients had more fever, dry cough, myalgia, and sore throat than probable (*p* < 0.05). Probable patients had more cerebrovascular (*p* = 0.041) and gastrointestinal system diseases (*p* = 0.003) than confirmed. Confirmed patients had more comorbidity related to the renal system than probable (*p* = <0.001). Confirmed patients had more surgical etiologies than probables (*p* < 0.001). Table 1 presents the demographic and clinical characteristics of the confirmed and probable patients. Bilateral ground-glass opacity (39.1%) and consolidation (28.1%) were the most common signs at chest CT in both groups. CT findings were not statistically different between the groups (*p* = 0.898) (Table 1).

**FIGURE 1:** Flowchart of confirmed and probable critically ill COVID-19 patients admitted to ICU. ICU: Intensive care unit.

**TABLE 1:** Demographic and clinical characteristics of confirmed and probable critically ill COVID-19 patients

The mean APACHE II score was 17.4 ± 8.2, GCS was 12.3 ± 3.9, and SOFA score was 5.9 ± 3.4 on ICU admission. There was no significant difference between groups in ICU severity scores and GCS. Confirmed patients were more tachypneic (*p* = 0.005) and more hypoxic (*p* = <0.001) than probable patients. Therefore, the percentage of inspired fractionated oxygen and the PEEP value was higher compared to probable patients (*p* < 0.005) (Table 2).

**TABLE 2:** Severity scores, vital signs, and measures of confirmed and probable patients on ICU admission

PaO_2_/FIO_2_ ratio was below 300 in 108 patients (84.4%). This ratio was lower in confirmed patients than probable (*p* = 0.001). Fifty-nine patients (46.1%) required endotracheal intubation, of which 28 were confirmed and 28 probable patients. There were no significant differences between the groups regarding requirement for low-flow oxygen, NIMV, and IMV. Confirmed critically ill patients were more likely to develop ARDS (98.4% vs. 59.7%) and HFOT when compared to probable patients (54.1% vs. 22.4%) (*p* < 0.001). Confirmed patients (n: 27, 44.2%) were mostly followed in the prone position (16.4%) (*p* = 0.001). Recruitment maneuvers were applied to 14 (10.9%) patients, eight were probable and six were confirmed. Tracheostomy was performed in two patients, one probable and one confirmed (Table 3). The most common PEEP was 8 (5-14) cm H_2_O in 23 mechanically ventilated patients.

**TABLE 3:** Treatments and complications of confirmed and probable critically ill COVID-19 patients

Probable critically ill patients were more likely to have pneumonia (83.6% vs. 41%), septic shock (36.7% vs. 27.9%), and vasopressor therapy (41.8% vs. 41%) compared with confirmed patients (*p* = 0.001, 0.039, and 0.004, respectively). The most used vasopressor was norepinephrine (n: 51 patients, 39.8%) and norepinephrine only use was more common in confirmed patients (n: 25 patients) (*p* = 0.004). Usage of steroid, Vitamin C use, and thromboprophylaxis was not statistically significantly different between the groups (Table 3). Out of 76 patients (59.4%) with AKI, 53 (86.9%) were confirmed and 23 (34.3%) were probable. AKI was more common in confirmed patients than probables, especially in Stage 3 (*p* < 0.001). RRT was performed in 30 of 76 patients with AKI; three patients received continuous RRT (CRRT), all of them were used in probable cases (Table 3). While DIC was more common in confirmed patients (19.7% vs. 16.4%), PTE and DVT were more common in probables (10.4% vs. 4.9% and 4.5% vs. 0%). One confirmed patient required extracorporeal membrane oxygenation (Table 3).

All critically ill patients received favipiravir therapy, one patient azithromycin, 9 patients (7%) hydroxychloroquine, and 2 patients (1.6%) oseltamivir for a maximum of 10 days. Fifteen patients (11.7%) convalescent plasma therapy, all of them were confirmed. Of the 5 patients (3.9%) who received tocilizumab, 4 (6.6%) were confirmed, and 1(1.5%) was probable.

Only 1 patient (0.8%) did not receive any antibiotic treatment. If necessary, empirical antibiotic therapy was revised according to results of microbiological culture during the ICU stay. Secondary bacterial infections were detected among 72 patients (56.3%) and more common in probable patients (62.1% vs. 50.8%).

Laboratory data including hemoglobin, fibrinogen, D-dimer, and CRP were significantly higher in confirmed patients when compared to probables. However, leukocytes, neutrophil, and total bilirubin were higher in probables (*p* = 0.03). There was no statistically significant difference between the groups for ferritin (Table 4). LDH (*p* = 0.007) and PCT (*p* = 0.11) were higher and thrombocyte (*p* = 0.027) was lower in the COVID-19 patients who died in the ICU compared to the survivors. PCT (*p* = 0.012) was higher and thrombocyte (*p* = 0.01) was lower in those who died in the hospital compared to the survivors. Overall, PCT (*p* = 0.027) and LDH (*p* = 0.032) were higher, lymphocyte (*p* = 0.043) and thrombocyte (*p* = 0.004) lower in non-survivors compared to survivors.

**TABLE 4:** Laboratory parameters of confirmed and probable critically Ill COVID-19 patients

While 81 patients (63.3%) were transferred to the ward, 52 patients (40.6%) were discharged from the hospital. The mean length of stay in ICU and hospital was 6.7 ± 6.2 and 15.3 ± 18 days. During the ICU admission, 21 confirmed and 26 probable patients died. The ICU mortality rate was 36.7%, hospital mortality rate was 41.4%, and overall mortality rate was 59.4%. Overall mortality was higher in COVID-19 patients with hypertension (*p* = 0.05), respiratory system (*p* = 0.001), and renal system diseases (*p* < 0.001). Overall mortality was higher in the confirmed group (52.6%) when compared to probables (47.4%) (*p* = 0.209) (Table 5).

**TABLE 5:** LOS and outcomes of confirmed and probable critically ill COVID-19 patients

## DISCUSSION

In this study, we admitted 128 confirmed and probable critically ill COVID-19 patients to the ICU during the normalization period. Confirmed patients were more hypoxemic, more tachypneic and had more fever, dry cough, myalgia, and sore throat than probable patients. Confirmed patients have more surgical etiology. Probable patients had more cerebrovascular and gastrointestinal system diseases than confirmed. We detected that ARDS, AKI, usage of HFOT-convalescent immune plasma, and prone position were more common in confirmed patients and confirmed patients had higher hemoglobin, CRP, D-dimer, and fibrinogen values. However, pneumonia, septic shock, and usage of vasopressor therapy were common in probable patients. Laboratory values including leukocytes, neutrophil, and total bilirubin were higher in probable patients. Overall mortality was higher in confirmed patients.

PCR is the most effective method to diagnose patients infected with COVID-19. Test performance is tied to disease prevalence [16,17]. The sensitivity is 80% and specificity is assumed to be 99% [18]. The diagnostic period begins 2 days before patients become symptomatic and extends to a highly variable period thereafter. In an estimated 20–40% of patients with few or no symptoms, it was difficult to determine the range of viral transmission and timing to detect a positive RT-PCR SARS-CoV-2 test [19,20]. Infected or symptomatic patients may have negative results due to many factors. These factors are as follows: Poor quality sample with little material, testing at early or late stage of infection, failure to process, and send the sample properly, technical reasons such as PCR inhibition or virus mutation, fluctuating distribution of the virus in symptomatic and asymptomatic cases [8]. Therefore, probable cases are considered to be patients with low viral load or in whom the range of viral transmission is difficult to detect. In our study, we could not perform the test during the viral transmission period to detect PCR positivity in our 67 probable patients.

We found that confirmed patients in the ICU had more surgical etiology. Because, during the normalization period, elective surgical procedures were continued uninterruptedly in our hospital. Hence, hospital and health care workers’ associated exposure increased. Nguyen et al. reported an increased risk of SARS-CoV-2 infection among frontline health care workers compared with the general population [21]. Front-line health care workers are at high risk of infection, contributing to further spread [22]. We think that long hospital stays and exposure to health care workers before and after the surgical procedure were associated with increased contact and transmission.

Dyspnea was reported in 75% of the patients on admission to the ICU. Fever, dry cough, myalgia, and sore throat were more common in confirmed patients than probables. Gong et al. showed that the classic triad (fever, dry cough, and dyspnea) of COVID-19 was more common in severe patients (42.7%) [23]. Viral load of COVID-19 has been shown to be associated with markers of inflammation and disease severity [24]. It can be said that PCR positivity is thought to be related to viral load and causes more viral infection-related symptoms.

The PaO_2_/FiO_2_ ratio corresponds to the severity of ARDS and it is correlated with increased mortality by the Berlin definition [13]. In our study, this ratio was lower in confirmed patients than probables. Because, viral load is higher in confirmed cases. The excess of viral load is associated with the severity of symptoms and disease [24,25]. Compared with probables (59.7%), confirmed patients (98.4%) were more likely to develop ARDS in our study. Huang et al. reported ARDS in 85% of patients admitted to ICU [3] and Yang et al. found in 67% [26]. Zhou et al. reported that ARDS was more observed in non-survivors [27]. We also found the incidence of ARDS to be high at a rate similar to other studies and we found that this rate was even higher in confirmed cases. We attribute the higher rate in confirmed cases to the high viral load and excess ACE2 receptor in the lungs. Compared to probables, confirmed critically ill patients received more HFOT because 70.5% of the confirmed patients had a P/F ratio of 200 or less. This ratio was lower in confirmed patients than probable (*p* = 0.001). This may indicate that confirmed patients have more severe and critical symptoms. Beduneau et al. presented their support for the use of HFOT as first-line therapy in severe patients in whom low-flow oxygen does not provide adequate respiratory support [28].

In our study, confirmed critically ill patients were followed more in the prone position compared to probables (45% vs. 16.9%). In the study of Mathews et al. including 2338 COVID-19 patients with moderate-to-severe ARDS, the early prone positioning was associated with lower hospital mortality compared without or later onset of prone positioning [29]. At present, with sufficient evidence, the prone position is a widely accepted recommended practice for the treatment of respiratory failure associated with COVID-19 [30,31]. However, cooperative patients should be in collaboration with health-care professionals for a prone position. In our study, the number of patients followed in the prone position was low due to the low number of collaborative patients.

COVID-19 may be characterized by sepsis secondary to viral infection. These causes can also be seen in septic shock, which causes severe organ dysfunction. In many published studies, the estimated prevalence of sepsis and septic shock ranges from 6.8 to 100% and 7.3 to 50 % [23,27]. In our study, we reported that 42 patients (32.8%) had septic shock which was more frequent among probables (37.3 %) when compared to confirmed patients (27.8%). Thus, the usage of vasopressor and inotropic therapy was also higher in probable patients. The frequency of pneumonia was higher in probables than confirmed patients. Sometimes, the causes of inflammation in COVID-19 could be multifactorial and participants without detectable plasma viremia also had elevated inflammatory markers [24]. Furthermore, there are sometimes delays in the treatment of probable patients with a lower viral load. We think that this may be related to the higher incidence of secondary complications to COVID-19.

COVID-19 affects multiple organs apart from the respiratory system; however, its renal manifestations are not clearly defined. In our study, 76 of total patients (59.4%) and 86.9% of confirmed patients had AKI. Many clinical trials have been reported that the incidence of AKI was 15-50% in critically ill COVID-19 patients [32-36]. We think that this high rate may be due to the higher expression of ACE2 in podocytes and proximal tubules of COVID-19 patients.

At this time, the use of therapeutic agents in the treatment of COVID-19 is controversial, as there are currently no randomized controlled trials [37]. All patients were given favipiravir and we administered azithromycin, hydroxychloroquine, and oseltamivir therapy among our patients. According to the Ministry of Health guideline, favipiravir was the only recommended antiviral treatment during the normalization period in our country. All patients who received convalescent immune plasma therapy were confirmed and tocilizumab was used more in confirmed patients than probables. Convalescent immune plasma therapy and anticytokine treatments are used in patients with COVID-19 PCR positivity as required by the health policy in our country [8].

Laboratory data including hemoglobin, D-dimer, CRP, and fibrinogen were significantly higher in confirmed critically ill patients compared to probables. However, leukocytes, neutrophil, and total bilirubin were higher in probables. In general, confirmed COVID-19 patients have higher CRP, D-dimer, fibrinogen, and leukocyte values [32]. No studies have been published that include such a comparison. It can be thought that PCR positivity triggering the inflammatory response may be related to elevated inflammatory laboratory values [26,27,33,38].

It has been reported that the mortality rates in critically ill patients with COVID-19 (not adjusted for severity) range from 0% to 85%, and this rate is between 41.6% and 50% in patients admitted to ICU [39,40]. In this study, the ICU mortality rate was 36.7%, hospital mortality rate was 41.4%, and overall mortality rate was 59.4%. Overall mortality was higher in confirmed critically ill COVID-19 patients. Mortality of confirmed cases were higher than prediction of APACHE-II scoring system. Higgins et al. also presented that APACHE appears to underestimate the ICU and hospital mortality [39]. Yang et al. also found a high mortality rate despite a mean APACHE score of 17 in COVID-19 patients [26]. Some patients may be well within the first 24 hours of data collection for the APACHE score and get worse after 24 hours. Therefore, their expected mortality may be underestimated by severity of disease captured during the first 24 hours after ICU admission. Zou et al. reported that APACHE II score was identified to be an effectively clinical tool to predict mortality in patients with COVID-19 and ≥17 serves as an early warning indicator of death. We presented that the mean APACHE II score was 17.4 as the previous studies [26,41]. However, we did not evaluate the association of the APACHE II score with mortality.

There are no clinical trials to compare probable and confirmed critically ill COVID-19 patients. Therefore, there were also some difficulties about discussing the results. Continuation of similar studies will help us in this regard. We think that comparing a larger number of confirmed and probable patients will provide us with updated and different information about the diagnosis, treatment, and management of COVID-19.

### Limitations

This study has some limitations. It was a retrospective study and had a small number of participants. It was conducted at a single center, which limits the generalizability of the results. The data were collected from the digital patient records. Not all laboratory tests were done in all patients.

## CONCLUSION

As a conclusion, our study indicates that critically ill confirmed COVID-19 patients had more end-organ failures including ARDS, AKI, and higher mortality. Complications and mortality rate are more common among confirmed COVID-19 patients admitted to ICU. The excess of viral load in confirmed patients admitted to ICU may be related to severity and adverse clinical outcomes. Mortality of confirmed cases was higher than prediction of APACHE-II scoring system. Due to the lack of data comparing clinical, laboratory, and radiological features of confirmed and probable cases, we think that similar clinical trials will provide us with updated information about the diagnosis, treatment, and management of COVID-19. Further investigation of the characteristics and differences of confirmed and probable COVID-19 patients is recommended in the future.

## References

[1] World Health Organization (2021). Coronavirus Disease (COVID-2019) Situation Reports.

[2] World Health Organization (2021). Coronavirus Disease (COVID-19) Outbreak.

[3] Huang C, Wang Y, Li X, Zhao J, Hu Y, Zhang L (2020). Clinical features of patients infected with 2019 novel Coronavirus in Wuhan, China. Lancet.

[4] Tan W, Zhao X, Ma X, Wang W, Niu P, Xu W (2020). A novel coronavirus genome identified in a cluster of pneumonia cases-Wuhan, China 2019-2020. China CDC Weekly.

[5] (2020). COVID-19 New Coronavirus Disease, Republic of Turkey, Ministry of Health.

[6] Wu Z, McGoogan JM (2020). Characteristics of and important lessons from the Coronavirus disease 2019 (COVID-19) outbreak in China:Summary of a report of 72314 cases from the Chinese center for disease control and prevention. JAMA.

[7] Falzone L, Musso N, Gattuso G, Bongiorno D, Palermo CI, Scalia G (2020). Sensitivity assessment of droplet digital PCR for SARS-CoV-2 detection. Int J Mol Med.

[8] COVID-19 (SARS-CoV-2 INFECTION) Guide (2020). Republic of Turkey, Ministry of Health, Ankara.

[9] World Health Organization (2020). Clinical Management of Severe Acute Respiratory Infection when Novel Coronavirus (2019-nCoV) Infection is Suspected:Interim Guidance.

[10] Alhazzani W, Moller MH, Arabi YM, Loeb M, Gong MN, Fan E (2020). Surviving sepsis campaign:Guidelines on the management of critically ill adults with Coronavirus disease 2019 (COVID-19). Intensive Care Med.

[11] Metlay JP, Waterer GW, Long AC, Anzueto A, Brozek J, Crothers K (2019). Diagnosis and treatment of adults with community-acquired pneumonia. An official clinical practice guideline of the American thoracic society and infectious diseases society of America. Am J Respir Crit Care Med.

[12] Kidney Disease:Improving Global Outcomes (KDIGO) Acute Kidney Injury Work Group (2012). KDIGO Clinical Practice Guideline for Acute Kidney Injury.

[13] Ranieri VM, Rubenfeld GD, Thompson BT, Fergoson ND, Caldwell E, ARDS Definition Task Force (2012). Acute respiratory distress syndrome:The Berlin definition. JAMA.

[14] McGonagle D, O'Donnell JS, Sharif K, Emery P, Bridgewood C (2020). Immune mechanisms of pulmonary intravascular coagulopathy in COVID-19 pneumonia. Lancet Rheumatol.

[15] Taylor FB, Toh CH, Hoots WK, Wada H, Levi M (2001). Scientific Subcommittee on Disseminated Intravascular Coagulation (DIC) of the International Society on Thrombosis and Haemostasis (ISTH). Towards definition, clinical and laboratory criteria, and a scoring system for disseminated intravascular coagulation. Thromb Haemost.

[16] Falzone L, Gattuso G, Tsatsakis A, Spandidos DA, Libra M (2021). Current and innovative methods for the diagnosis of COVID-19 infection (review). Int J Mol Med.

[17] Dramé M, Tabue Teguo M, Proye E, Hequet F, Hentzien M, Kanagaratnam L (2020). Should RT-PCR be considered a gold standard in the diagnosis of COVID-19?. J Med Virol.

[18] (2020). CDC 2019-Novel Coronavirus (2019-nCoV) Real-Time RT-PCR Diagnostic Panel Instructions for Use.

[19] Murad D, Chandrasekaran S, Pillai A, Garner OB, Denny CT (2021). SARS-CoV-2 infection detection by PCR and serologic testing in clinical practice. J Clin Microbiol.

[20] Mizumoto K, Kagaya K, Zarebski A, Chowell G (2020). Estimating the asymptomatic proportion of Coronavirus disease 2019 (COVID-19) cases on board the Diamond Princess cruise ship, Yokohama, Japan, 2020. Euro Surveill.

[21] Nguyen LH, Drew DA, Graham MS, Joshi AD, Guo CG, Ma W (2020). Risk of COVID-19 among front-line health-care workers and the general community:A prospective cohort study. Lancet Public Health.

[22] Black JRM, Bailey C, Przewrocka J, Dijkstra KK, Swanton C (2020). COVID-19:The case for health-care worker screening to prevent hospital transmission. Lancet.

[23] Gong X, Kang S, Guo X, Li Y, Gao H, Yuan Y (2021). Associated risk factors with disease severity and antiviral drug therapy in patients with COVID-19. BMC Infect Dis.

[24] Fajnzylber J, Regan J, Coxen K, Corry H, Wong C, Rosenthal A (2020). SARS-CoV-2 viral load is associated with increased disease severity and mortality. Nat Commun.

[25] Pujadas E, Chaudhry F, McBride R, Richter F, Zhao S, Wajnberg A (2020). SARS-CoV-2 viral load predicts COVID-19 mortality. Lancet Respir Med.

[26] Yang X, Yu Y, Xu J, Shu H, Xia J, Liu H (2020). Clinical course and outcomes of critically ill patients with SARS-CoV-2 pneumonia in Wuhan, China:A single-centered, retrospective, observational study. Lancet Respir Med.

[27] Zhou F, Yu T, Du R, Fan G, Liu Y, Liu Z (2020). Clinical course and risk factors for mortality of adult inpatients with COVID-19 in Wuhan, China:A retrospective cohort study. Lancet.

[28] Beduneau G, Boyer D, Guitard PG, Gouin P, Carpentier D, Grange S (2021). Covid-19 severe hypoxemic pneumonia:A clinical experience using high-flow nasal oxygen therapy as first-line management. Respir Med Res.

[29] Mathews KS, Soh H, Shaefi S, Wang W, Bose S, Coca S (2021). Prone positioning and survival in mechanically ventilated patients with Coronavirus disease 2019-related respiratory failure. Crit Care Med.

[30] Dembinski R (2021). Prone positioning in Coronavirus disease 2019:Just do it!. Crit Care Med.

[31] Sun Q, Qiu H, Huang M, Yang Y (2020). Lower mortality of COVID-19 by early recognition and intervention:Experience from Jiangsu province. Ann Intensive Care.

[32] Gómez-Escobar LG, Hoffman KL, Choi JJ, Borczuk A, Salvatore S, Alvarez-Mulett SL (2021). Cytokine signatures of end organ injury in COVID-19. Sci Rep.

[33] Richardson S, Hirsch JS, Narasimhan M, Crawford JM, McGinn T, Davidson KW (2020). Presenting characteristics, comorbidities, and outcomes among 5700 patients hospitalized with COVID19 in the New York city area. J Am Med Assoc.

[34] Gabarre P, Dumas G, Dupont T, Darmon M, Azoulay E, Zafrani L (2020). Acute kidney injury in critically ill patients with COVID-19. Intensive Care Med.

[35] Zamoner W, Santos CA, Magalhães LE, de Oliveira PG, Balbi AL, Ponce D (2021). Acute kidney injury in COVID-19:90 Days of the pandemic in a Brazilian public hospital. Front Med (Lausanne).

[36] Cheng Y, Zhang N, Luo R, Zhang M, Wang Z, Dong L (2021). Risk factors and outcomes of acute kidney injury in critically Ill patients with Coronavirus disease 2019. Kidney Dis (Basel).

[37] Sweeney DA, Benson CA, Kalil AC (2021). Convalescent plasma and Coronavirus disease 2019:Time for reassessment. Crit Care Med.

[38] Wang D, Hu B, Hu C, Zhu F, Liu X, Zhang J (2020). Clinical characteristics of 138 hospitalized patients with 2019 novel Coronavirus-infected pneumonia in Wuhan, China. JAMA.

[39] Higgins TL, Stark MM, Henson KN, Freeseman-Freeman L (2021). Coronavirus disease 2019 ICU patients have higher-than-expected acute physiology and chronic health evaluation-adjusted mortality and length of stay than viral pneumonia ICU patients. Crit Care Med.

[40] Armstrong RA, Kane AD, Cook TM (2020). Outcomes from intensive care in patients with COVID-19:A systematic review and meta-analysis of observational studies. Anaesthesia.

[41] Zou X, Li S, Fang M, Hu M, Bian Y, Ling J (2020). Acute physiology and chronic health evaluation II score as a predictor of hospital mortality in patients of Coronavirus disease 2019. Crit Care Med.

